The article "Triptolide inhibits oxidative stress and inflammation via the microRNA-155-5p/brain-derived neurotrophic factor to reduce podocyte injury in mice with diabetic nephropathy" was retracted in 2026. Reasons: concerns about the data; concerns about the results or conclusions.

# Triptolide inhibits oxidative stress and inflammation via the microRNA-155-5p/brain-derived neurotrophic factor to reduce podocyte injury in mice with diabetic nephropathy

**DOI:** 10.1080/21655979.2022.2067293

**Published:** 2022-05-21

**Authors:** Jian Gao, Zheng Liang, Fei Zhao, Xiaojing Liu, Ning Ma

**Affiliations:** The First Department of Nephrology, Cangzhou Central Hospital, Cangzhou, Hebei, China

**Keywords:** Diabetic nephropathy, podocytes, triptolide, miR-155-5p, brain-derived neurotrophic factor, oxidative stress, inflammation

## Abstract

Diabetic nephropathy (DN) is a complication of diabetes. This study sought to explore the mechanism of triptolide (TP) in podocyte injury in DN. DN mice were induced by high-fat diet&streptozocin and treated with TP. Fasting blood glucose, 24 h urine microalbumin (UMA), the pathological changes of renal tissues, and ultrastructure of renal podocytes were observed. Podocytes (MPC5) were induced by high-glucose (HG) *in vitro* and treated with TP or microRNA (miR)-155-5p mimics, with Irbesartan as positive control. Reactive oxygen species (ROS) and levels of oxidative stress (OS) and inflammatory factors in MPC5 were detected. The levels of miR-155-5p, podocyte marker protein Nephrin, and inflammatory factors in mice and MPC5 were detected. The targeting relationship between miR-155-5p and brain-derived neurotrophic factor (BDNF) was verified. The expression levels of BDNF were detected. miR-155-5p mimics and overexpressed (oe)-BDNF plasmids were co-transfected into mouse podocytes treated with HG and TP. TP reduced fasting glucose and 24 h UMA of DN mice, alleviated the pathological damage and podocyte injury, up-regulated Nephrin level, and down-regulated miR-155-5p. TP down-regulated the high expression of miR-155-5p in HG-induced MPC5 cells and inhibited HG-induced OS and inflammatory injury, and the improvement effect of TP was better than Irbesartan. Overexpression of miR-155-5p reversed the protective effect of TP on injured mouse podocytes. miR-155-5p targeted BDNF. oe-BDNF reversed the inhibitory effect of oe-miR-155-5p on TP protection on podocyte injury in mice. Overall, TP up-regulated BDNF by inhibiting miR-155-5p, thus inhibiting OS and inflammatory damage and alleviating podocyte injury in DN mice.

## Introduction

Diabetic Nephropathy (DN) is one of the major microvascular complications of diabetes[1]. With the development of the economy and the improvement of people’s living standards, the global prevalence of diabetes is increasing, and the incidence of DN is also on the rise [2]. Despite the complicated pathogenesis of DN, podocyte injury has been identified to play essential roles [3]. Structural changes or damage to podocytes are associated with kidney injury, resulting in proteinuria and severe renal insufficiency, and eventually leading to DN [4]. Furthermore, impaired podocytes lead to impaired selective glomerular filtration and contribute to the formation of proteinuria [5]. Meanwhile, the production of reactive oxygen species (ROS) induced by persistent hyperglycemia will inevitably damage the antioxidant defense system, and trigger oxidative stress (OS) and inflammatory responses [6]. In consequence, it is of great significance to study the mechanism of podocyte injury in DN.

Triptolide (TP), extracted from Tripterygium wilfordii, has extensive biological functions, such as immunosuppression, anti-inflammatory, antifertility, and neuroprotection [7]. TP has also been reported to have protective effects on DN [8]. TP can significantly alleviate proteinuria and podocyte damage in animal models of DN [9]. Importantly, TP stabilizes the podocyte cytoskeleton and protects against podocyte diseases, including microvariant diseases, focal glomerulosclerosis, and membranous nephropathy [8]. However, the mechanism of TP in the treatment of DN has not been fully elucidated.

MicroRNAs (miRNAs) are small noncoding RNAs that modulate gene expression by down-regulating mRNA levels or directly inhibiting gene translation [10]. It has been reported that miRNAs are closely involved in the regulatory process of DN [11]. For instance, miR-494-3p and miR-574-5p can regulate the specific expression of complement C7 in mesangial cells and serve as potential diagnostic biomarkers for DN [12]. miR-188-3p disrupts germacrone-mediated podocyte protection in a DN mouse model in type I diabetes by triggering mitochondrial damage [13]. Some researchers have found that miR-155-5p is overexpressed in the serum of DN patients, and miR-155-5p may become a potential diagnostic marker for DN [14,15]. Another researcher found that dihydromyrrhetin promotes autophagy and alleviates renal interstitial fibrosis in DN by regulating the miR-155-5p/PTEN axis [16]. Through literature review, we learned that the p53/miR-155-5p/SIRT axis can relieve renal tubule injury in DN [17]. Recently, it has also been reported that inhibition of miR-155-5p protects renal tubular epithelial cells from high glucose (HG)-induced inflammation, OS, apoptosis, and lipid accumulation [18]. These studies suggest that miR-155-5p may be an important target for the treatment of DN.

Brain-derived neurotrophic factor (BDNF) is closely involved in the repair of DN podocytes and is widely expressed in podocytes [19]. Meanwhile, BDNF has extensively been documented in the regulation of inflammatory factors, fibrosis, and renal function in DN mice [20] and cellular OS [21,22] in other diseases. However, it has not been reported that TP inhibits podocyte injury by regulating the miR-155-5p/BDNF pathway. Therefore, this study was to explore the therapeutic effect of TP on DN, hoping to provide new insights into the pathogenesis and treatment of DN.

## Materials and methods

### Ethics statements

The animal experiments were approved by the animal Ethics Committee of Cangzhou Central Hospital (Approval number: 20,191,015), and the pain and number of experimental animals were minimized during the experiment.

### Animal treatment and grouping

A total of 36 C57BL/6 J male mice (6 weeks old, weighing 16 ± 2 g) were provided by Vital River Laboratory Animal Technology (Beijing, China). Free diet and drinking water were provided, and the mice were kept in separate cages at 22 ± 1 under the conditions of 12 h light and dark cycles with an air humidity of 55–65%. After 1 week of adaptive feeding, 10 mice were randomized to the normal control (NC) group and fed a normal diet. As previously described [23], the remaining 26 mice were fed a high-fat diet (HFD) for 8 weeks and then given a single intraperitoneal injection of streptozocin (STZ) (30 mg/Kg), which was dissolved in sodium citrate buffer. Meanwhile, the mice in the NC group were injected with an equal amount of sodium citrate buffer. Then, 72 h after STZ injection, the fasting glucose level of mice was measured, and the 24 h-urine samples in the metabolic cage were collected to detect 24 h urinary microalbumin (UMA). Mice with the fasting glucose ≥16.7 mmol/L and 24 h UMA higher than NC mice were included in the DN group (5 mice that did not meet the requirements and 1 mouse that died were excluded, and 20 mice were included in the DN group finally). Next, 10 DN mice were randomized to the TP treatment group (DN + TP group) and treated with TP by gavage (50 ug/kg/d, D0777-20 mg, HPLC > 99%, Baoman Biological Technology, Shanghai, China). The remaining 10 mice were given an equal amount of normal saline containing 0.4% dimethyl sulfoxide (FT-67-68-5, Fantai Biological Technology, Shanghai, China) by gavage for 12 weeks. TP was dissolved in dimethyl sulfoxide and diluted with normal saline. The dosage and treatment were adjusted according to the literature [8,10,11].

### Detection of fasting glucose and 24 h UMA in mice

After continuous treatment with TP for 12 weeks, 24 h urine samples of all mice in the treatment groups were collected in the metabolic cage on the day before index detection, and the fasting glucose and 24 h UMA were detected in the morning of the next day [24]. The fasting glucose level of the mice was determined by the blood glucose detection kits (CS-M100278, Chuntest Biotechnology, Shanghai, China), and the 24 h UMA was determined by the mouse urinary albumin enzyme-linked immunosorbent assay (ELISA) kit (EY-M98316, Yiyan Biotechnology, Shanghai, China). The operation strictly followed the instructions of the kit.

### Hematoxylin-eosin (HE) staining

Following previous work [25], after the measurement of fasting glucose and 24 h UMA, the mice were euthanized with sodium pentobarbital (30 mg/kg body weight), and the abdominal cavity of mice was opened. Then, the left and right kidneys of mice were removed, and the residual blood in the kidneys was washed with pre-cooled normal saline at 4°C. The left kidney was cut in half longitudinally in the middle and fixed in the refrigerator at 4°C for 24 h with 10% paraformaldehyde. The kidney tissues were embedded in paraffin and made into paraffin sections with a thickness of 3 μm. The prepared sections were routinely dewaxed, hydrated, stained in hematoxylin staining solution (G1140, Solarbio, Beijing, China) for 2 min, and then rinsed with tap water. After differentiation with 1% hydrochloric acid ethanol for 3–5 seconds, the sections were washed with tap water again and treated with 1% ammonia for 3–5 s to return to blue. Following washing with tap water, the sections were restained with eosin for 1 min, washed with tap water, dehydrated with gradient ethanol, cleared with xylene, and then sealed with neutral gum. The pathological changes of mouse kidney tissues were observed under a light microscope (Olympus, Tokyo, Japan).

### Transmission electron microscope (TEM) observation

As previously described [8], the cortical tissue of the right kidney of mice was collected and cut into 1 mm^3^ with the blade. The tissues were fixed with 3.75% glutaraldehyde and 1% osmic acid, embedded with epoxy resin, stained with uranyl acetate and citric acid. The ultrastructural changes of mouse podocytes were observed under the TEM (Olympus). Reverse transcription quantitative polymerase chain reaction (RT-qPCR) and Western blot (WB) were utilized to detect the expression in residual cortical tissues of the right kidney.

### Cell culture

Following previous work [26], conditionally immortalized mouse podocytes (MPC5) provided by the Cell Bank of the Chinese Academy of Sciences in Shanghai were cultured in RPMI 1640 medium (Gibco, MA, USA) supplemented with 10% fetal bovine serum and 1% penicillin/streptomycin (all purchased from Fantai Biotech) in an incubator with 5% CO_2_ at constant 37°C.

### Cell grouping and transfection

According to the literature [26], after the recovery, passage, and differentiation of MPC5 cells, the cells were grouped as follows: (1) NG group (Normal glucose), MPC5 cells were cultured in RPMI 1640 medium supplemented with 5.5 mM glucose for 48 h; (2) HG group, MPC5 cells were cultured with 25 mM glucose in RPMI 1640 medium for 48 h, and the concentration of HG was determined as per the reference [27]; (3) HG + TP group, MPC5 cells were cultured with 25 mM glucose and 10 uM TP in RPMI 1640 medium for 48 h, and the administration method and dosage of TP were referred to a previous study [10]. (4) HG + IRB group, MPC5 cells were cultured in RPMI 1640 medium supplemented with 25 mM glucose and 10 uM irbesartan for 48 h, with irbesartan used as a positive control. The administration method and dosage were referred to previous studies [28,29]. (5) HG + TP + miR-NC group, 25 mM glucose and 10 uM TP were added into the RPMI 1640 medium, and MPC5 cells were transfected with negative control of miR-155-5p and cultured in the medium for 48 h. (6) HG + TP + miR-155-5p group, 25 mM glucose and 10 uM TP were added into RPMI 1640 medium, and MPC5 cells were transfected with miR-155-5p mimics and cultured in the medium for 48 h. (7) HG + TP + miR-155-5p + overexpression (oe)-NC group, 25 mM glucose and 10 uM TP were added into the RPMI 1640 medium, and MPC5 cells were co-transfected with miR-155-5p mimics and oe-NC empty plasmid and cultured in the medium for 48 h. (8) HG + TP+ miR-155-5p + oe-BDNF group, 25 mM glucose and 10 uM TP were added into RPMI 1640 medium, MPC5 cells were co-transfected with miR-155-5p mimics and oe-BDNF plasmids, and cultured in the medium for 48 h. The overexpressed miR-155-5p and BDNF plasmids and their corresponding controls were designed and synthesized by Yingbio Technology (Shanghai, China). Transfection experiments were performed using Lipofectamine 2000 (Invitrogen, CA, USA). After 48-h culture, the MPC5 cells from each group were collected for subsequent experimentation.

### Reactive oxygen species (ROS) detection

Following previous work [30], intracellular ROS levels were determined by the 2,7 dichlorofluorescin-diacetic acid determination method (DCFH-DA, Solarbio). Briefly, the collected cells were prepared into cell suspension using phosphate buffer saline (PBS) and seeded into 6-well plates at 5000 cells/well. DCFH-DA solution with a final concentration of 5 mM was added into the suspension and incubated at 37°C for 30 min. After washing with PBS, the fluorescence intensity was detected using a fluorescence microscope (IX70, Olympus), and the emission wavelength was set at 530 nm and excitation wavelength was set at 485 nm.

### Detection of OS

As previously described [31], MPC5 cells in each group were collected, and the activities of malondialdehyde (MDA) (A003-1-1), superoxide dismutase (SOD) (A001-1-2), and glutathione (GSH) (A005-1-2) were detected using ELISA kits (Jiancheng Bioengineering Institute, Nanjing, China). The operation strictly followed the instructions of the kit.

### Detection of inflammatory-related factors

Following previous work [31], MPC5 cells in each group were collected, and the levels of inflammatory cytokines such as interleukin-1β (IL-1β) (H002), interleukin (IL)-6 (H007-1-1), tumor necrosis factor (TNF)-α (H052-1), and IL-4 (H005) were detected by ELISA kits (Jiancheng Biological). The operation strictly followed the instructions of the kit.

### RT-qPCR

As previously described [32], total RNA was extracted from mouse renal cortex tissues or cells using the total RNA extraction kit (DP420, Tiangen Biochemical Technology, Beijing, China). The RNA was reverse transcribed to cDNA using a Taqman® Micro RNA Reverse Transcription Reagents kit (Invitrogen). The RT-qPCR was performed using ABI Prism 7300 system (Applied Biosystems, USA) under the following reaction procedures: pre-denaturation at 95°C for 10 min, and 35 cycles of denaturation at 90°C for 10 s, annealing at 63°C for 15 s, and extension at 72°C for 30 s. The 2-ΔΔCT method was used to calculate the relative levels of the target genes, with U6 and β-actin as the internal references of miR-155-5p and BDNF, and then the data were normalized. The primer sequences for each gene were synthesized by Beyotime (Shanghai, China), as shown in Table 1.

**Table 1.** Primer sequence

Gene	Forward 5'-3'	Reverse 5'-3'
*miR-155-5p*	CGCGTGGGGATAGTGTTAATC	AGTGCAGGGTCCGAGGTATT
*BDNF*	AGCTGAGCGTGTGTGACAGTAT	CCGAACATACGATTGGGTAGTT
*U6*	GCTTCGGCAGCACATATACTAAAAT	CGCTTCACGAATTTGCGTGTCAT
*β-actin*	GCCATGTACGTAGCCATCCA	GAACCGCTCATTGCCGATAG

### WB detection

As mentioned previously [30], total protein was extracted from renal cortex tissues or cells from each group using Radio Immunoprecipitation Assay (RIPA) lysate (AR0105, Hengfei Biotechnology, Shanghai, China). After the protein concentration was detected with the bicinchoninic acid assay kit (701,780–480, Cayman, USA), the protein was isolated using 10% sodium dodecyl sulfate-polyacrylamide gel electrophoresis and transferred to the polyvinylidene fluoride membranes. The membranes were blocked with 5% skim milk for 1 h and incubated overnight with rabbit primary antibodies anti-nephrin (1/500, ab216692, Abcam, 136 kDa), anti-BDNF (1/1000, ab189494, Abcam, 110 kDa), anti-IL-1β (1/1000, ab234437, Abcam, 31k Da), anti-IL-6 (1/1000, ab208113, Abcam, 23 kDa), anti-TNF-α (1/1000, ab255275, Abcam, 25 kDa), anti-IL-4 (1/500, ab84269, Abcam, 17 kDa), and anti-β-actin (1/20,000, ab179467, Abcam, 42 kDa) at 4°C. After washing, the membrane was added with the HRP-labeled goat anti-rabbit secondary antibody IgG H&L (1:2000, ab136636, Abcam) at room temperature for 1 h, and then developed using enhanced chemiluminescence, and photographed. Image-Pro Plus 6.0 (Media Cybernetics, USA) was used to analyze the gray values of the bands, with β-actin as the internal reference.

### Dual-luciferase reporter assay

Following previous work [30], the targeted binding sites between miR-155-5p and BDNF were predicted using the online bioinformatics software TargetScan (http://www. Targetscan.org). The pGL3 dual-luciferase reporter plasmid vectors of BDNF-3’UTR wild-type (BDNF-WT) and mutant (BDNF-MUT) were designed and constructed by R&S Biotechnology (Shanghai, China). BDNF-WT or BDNF-MUT plasmid vectors were co-transfected into MPC5 cells cultured in normal glucose with miR-155-5p mimics or miR-155-5p NC. At 48 h after transfection, the ratio of firefly luciferase to Renilla luciferase (firefly luciferase/Renilla luciferase) was determined as the relative expression of luciferase.

### Statistical analysis

SPSS 19.0 software (IBM Corp. Armonk, NY, USA) was employed for statistical analyses. Data were expressed as mean ± standard deviation (SD). The Mann–Whitney *U* test was used for data comparison between two groups and Kruskal–Wallis univariate analysis of variance (ANOVA) (k samples) test was used for data comparison among multiple groups. *P* was obtained from a bilateral test, and a value of *P* < 0.05 was regarded significant difference.

## Results

Previous studies have shown that TP can reduce proteinuria and podocyte injury in DN animal models [8,9,33], but its specific mechanism has not been fully elucidated. miR-155-5p is one of the reasons for the increased secretion of inflammatory factors in renal tissue of DN, as well as one of the potential markers of DN [14,18]. At animal and cell levels, our study confirmed that TP up-regulated the level of BDNF by inhibiting the expression of miR-155-5p, and protected DN by inhibiting OS and inflammatory injury in renal tissues or podocytes of DN. Our findings provide a new theoretical reference for TP as a potential therapeutic agent for DN and further verify that miR-155-5p may be a new target for DN treatment.

### TP ameliorated DN and reduced podocyte injury in mice

To explore the mechanism of TP on DN, we established the DN mouse model by HFD feeding combined with STZ injection *in vivo*. The fasting glucose values ≥ 16.7 mmol/L for two consecutive times and 24 h UMA was higher than the NC group, which were used as the inclusion criteria of DN mice (Figure 1a,b, *P* < 0.01). After successful modeling, the DN mice were treated with TP for 12 weeks. Next, we tested the fasting glucose and 24 h UMA in different groups and found that the fasting glucose and 24 h UMA in mice were reduced after TP treatment (Figure 1a,b, *P* < 0.01). The morphological changes of renal tissues of mice in different groups were observed using HE staining, which showed that the structure of renal glomeruli and tubules was clear, the morphology was regular, and there was no obvious pathological change in the NC group, while the volume of renal glomeruli and tubules was enlarged, the structure was disordered and deformed in DN mice. After TP treatment, the morphological changes were improved (Figure 1c). Subsequently, we observed the morphological changes in mouse kidney podocyte by TEM and found that there were no significant pathological changes in podocytes in the NC group, while the podocyte in the DN group was fused, the number of podocyte slits was reduced, and the hiatus membrane slit diaphragms were disappeared. After TP treatment, the pathological changes of podocytes were improved (Figure 1c). We further detected the level of Nephrin, a marker protein in mouse podocytes, by WB, and found that compared with the NC group, Nephrin in the DN group was decreased and increased after TP treatment (Figure 1d). These results suggest that TP can improve DN and reduce podocyte damage in mice.

**Figure 1.** TP ameliorated DN and reduced podocyte injury in mice. The DN mouse model was induced by HFD feeding combined with injection of STZ *in vivo*, and treated with TP for 12 weeks. A: fasting glucose value of mice detected using kits B: 24 h UMA in mice; C: HE staining was used to observe the pathological changes of renal tissues and transmission electron microscopy was used to observe the ultrastructural changes of the podocyte in the renal cortex; D: WB was used to detect the level of Nephrin, a marker in renal podococytes of mice; Measurement data were expressed as mean ± standard deviation, N = 10, Kruskal–Wallis univariate ANOVA (k samples) test was used for data comparison among multiple groups. *P* value was obtained from a bilateral test, ** P < 0.01, *** P < 0.001.

### *TP inhibited miR-155-5p expression* in vitro *and* in vivo

Some researchers have reported the overexpression of miR-155-5p in the serum or plasma of DN patients [14,15]. To explore whether TP affects the miR-155-5p expression, we measured the miR-155-5p expression in kidney tissues of mice in different groups by RT-qPCR and found that miR-155-5p was overexpressed in kidney tissues of mice in the DN group, while TP could inhibit its expression (Figure 2a, all *P* < 0.01). In addition, we induced podocyte injury by HG *in vitro* experiments and intervened with TP, and detected the level of miR-155-5p by RT-qPCR. It was found that miR-155-5p was up-regulated in injured mouse podocytes induced by HG but inhibited by TP treatment (Figure 2b, all *P* < 0.01). In short, TP could inhibit miR-155-5p *in vivo* and *in vitro*.

**Figure 2.** TP inhibited the expression of miR-155-5p in mouse podocytes *in vitro* and *in vivo. In vivo*, the DN mouse model was induced by HFD feeding combined with STZ injection, and treated with TP for 12 weeks. *In vitro*, podocyte injury was induced by HG and podocytes were treated with TP for 48 h. A: The level of miR-155-5p in the kidney tissues of mice was detected by RT-qPCR; B: The level of miR-155-5p in mouse podocytes was detected by RT-qPCR; Measurement data were expressed as mean ± standard deviation, N = 10, the cell experiment was independently repeated 3 times. Kruskal-Wallis univariate ANOVA (k samples) test was used for data comparison among multiple groups. *P* value was obtained from a bilateral test, ** *P* < 0.01, *** *P* < 0.001.

### TP alleviated OS and inflammatory injury in MPC5 cells induced by HG by inhibiting miR-155-5p

Studies have shown that OS in DN is strongly associated with the imbalance of inflammatory factors [1,2,34]. Meanwhile, several studies have shown that TP has anti-effects on OS and inflammation [35–37]. We speculated that the protective effect of TP on DN may be related to OS and inflammation. Hence, the ROS levels in mouse podocytes MPC5 were quantitatively determined by DCFH-DA kits and fluorescence microscope, and the OS-related oxidase levels such as MDA, SOD, and GSH, as well as inflammation-related factors IL-1β, IL-6, TNF-α, and IL-4 were examined by ELISA kits. The results elicited that the ROS and MDA levels were increased in the HG group relative to the NG group, while SOD and GSH levels were decreased; after the intervention of TP, the ROS and MDA levels were decreased, while SOD and GSH levels were increased; the OS level of MPC5 cells in the HG + IRB group was also improved, but the effect of TP treatment was better (Figure 3a-d, all *P* < 0.05). Compared with the NG group, IL-1β, IL-6, and TNF-α were up-regulated, while IL-4 was down-regulated in the HG group; after the intervention of TP, IL-1β, IL-6, and TNF-α were down-regulated, while IL-4 was up-regulated; the imbalance of inflammatory factors in MPC5 cells in the HG + IRB group was also improved, but the effect of TP treatment was better (Figure 3e-h, all *P* < 0.05). Subsequently, we further detected the protein levels of IL-1β, IL-6, TNF-α, and IL-4 by WB, and the results were consistent with the trend of ELISA (Figure 3i). Briefly, TP can inhibit OS and inflammatory injury of mouse podocytes induced by HG.

**Figure 3.** TP alleviated oxidative stress and inflammatory damage in MPC5 cells induced by HG based on miR-155-5p. The podocyte injury was induced by HG and podocytes were treated with TP. Mouse podocytes treated with HG and TP were transfected with miR-155-5p mimics to increase the expression of miR-155-5p. After 48 h of treatment, relevant tests were performed. A: The ROS levels in mouse podocytes were detected by DCFH-DA kits. B-D: The levels of oxidative stress-related enzymes such as MDA, SOD, and GSH in MPC5 cells were detected by ELISA kits. E-H: The levels of Il-1 β, IL-6, TNF-α, and IL-4 in MPC5 cells were detected by ELISA kits; I: The protein levels of IL-1β, IL-6, TNF-α, and IL-4 in MPC5 cells were detected by WB. J: The level of miR-155-5p in mouse podocytes was detected by RT-qPCR; The value of miR-155-5p in Figure J was consistent with that in Figure 2b; Measurement data were expressed as mean ± standard deviation, the cell experiment was independently repeated 3 times. Kruskal-Wallis univariate ANOVA (k samples) test was used for data comparison among multiple groups. *P* value was obtained from a bilateral test, * *P* < 0.05, ** *P* < 0.01, *** *P* < 0.001.

To explore the role of miR-155-5p in TP protecting podocytes from injury, we transfected miR-155-5p mimics into mouse podocytes MPC5 after the combined intervention with HG and TP. RT-qPCR uncovered that the cells were successfully transfected (Figure 3j, p < 0.001). We then tested the indicators of OS and inflammation-related factors in MPC5 cells again and illustrated that overexpression of miR-155-5p reversed the protective effect of TP on injured mouse podocytes (Figure 3a-i, all *P* < 0.05). These results suggest that TP may reduce OS and inflammatory injury in MPC5 cells induced by HG based on miR-155-5p.

### miR-155-5p targeted BDNF

To explore the downstream target genes regulated by miR-155-5p, we first predicted 8 downstream potential target genes including BDNF by analyzing the intersection of 3 different bioinformatics websites (Targetscan, StarBase, and miRDB) (Figure 4a). Further reports suggested that BDNF was one of the important factors regulating OS and inflammation [21,22]. Meanwhile, BDNF was also reported to be involved in the regulation of DN [19]. Through the online bioinformatics website TagetScan, we predicted that there were targeted binding sites between the 3’UTR of BDNF and miR-155-5p (Figure 4b). We thus speculated the involvement of miR-155-5p in the regulation of OS and inflammatory factors in podocyte injury by targeting BDNF. The pGL3 plasmid vectors of BDNF-WT and BDNF-MUT were constructed and co-transfected into MPC5 cells with miR-155-5p mimics or miR-155-5p NC, respectively. At 48 h after transfection, the luciferase relative expression was measured. It was observed that the fluorescence intensity of MPC5 cells co-transfected with miR-155-5p mimics was lowered in the BDNF-WT group, while there was no significant difference in the MUT group, which demonstrated the presence of targeted binding sites between miR-155-5p and BDNF (Figure 4c, p< 0.001). Furthermore, we detected the levels of BDNF in different groups *in vitro* and *in vivo* by RT-qPCR and WB. *In vivo*, BDNF was down-regulated in the DN group compared with the NC group, while its expression was up-regulated after TP treatment (Figure 4d, all *P* < 0.01). I*n vitro*, relative to the NG group, BDNF was down-regulated in the HG group, up-regulated after TP treatment, and down-regulated again after treatment with miR-155-5p mimics (Figure 4e, all *P* < 0.01). Briefly, miR-155-5p targeted BDNF.

**Figure 4.** miR-155-5p targeted BDNF. A: The downstream target genes of miR-155-5p were analyzed by bioinformatics website Targetscan, StarBase, and miRDB. B: The bioinformatics software TargetScan predicted the targeted binding sites of miR-155-5p and BDNF; C: Dual-luciferase assay was used to detect the targeted binding sites of miR-155-5p and BDNF; D: The expression of BDNF in mice was detected by RT-qPCR and WB. E: The BDNF expression in mouse podocytes was detected by RT-qPCR and WB. Measurement data were expressed as mean ± standard deviation, N = 10, the cell experiment was independently repeated 3 times. Mann-Whitney U test was used for data comparison between two groups and Kruskal-Wallis univariate ANOVA (k samples) test was used for data comparison among multiple groups. *P* value was obtained from a bilateral test, ** *P* < 0.01, *** *P* < 0.001.

### TP protected against HG-induced podocytes injury through the miR-155-5p/BDNF axis

To further figure out the role of BDNF in OS and inflammatory injury of mouse podocytes, we co-transfected miR-155-5p mimics and BDNF overexpression plasmids into MPC5 cells co-interfered with HG and TP. The level of BDNF was detected by RT-qPCR and WB, which manifested that BDNF was successfully overexpressed (Figure 5a, all *P* < 0.001). We further examined the ROS, SOD, MDA, and GSH and the levels of IL-1β, IL-6, TNF-α, and IL-4 in MPC5 cells. It was unraveled that overexpression of BDNF alleviated OS and inflammatory injury, and partially restored the inhibition of the protective effect of TP by overexpression of miR-155-5P (Figure 5b-j, all *P* < 0.01). Conjointly, TP up-regulated BDNF levels by inhibiting miR-155-5p, thus inhibiting OS and inflammatory injury and alleviating mouse podocyte injury induced by HG.

**Figure 5.** Overexpression of BDNF antagonized the inhibition of overexpression of miR-155-5p on the protective effect of TP on MPC5 cell injury. The miR-155-5p mimics and overexpressed BDNF plasmid were co-transfected into MPC5 cells with HG and TP combined intervention, and related detection was performed 48 h after transfection. A: The level of BDNF in MPC5 cells was detected by RT-qPCR and WB. B: The ROS levels in MPC5 cells were detected by DCFH-DA kit; C-E: The levels of oxidative stress-related enzymes such as MDA, SOD, and GSH in MPC5 cells were detected by ELISA kits. F-I: The levels of IL-1β, IL-6, TNF-α, and IL-4 in MPC5 cells were detected by ELISA kits. J: The protein levels of IL-1β, IL-6, TNF-α, and IL-4 in MPC5 cells were detected by WB. The mRNA value of BDNF in Figure A was consistent with that in Figure 4e; Measurement data were expressed as mean ± standard deviation, and Kruskal-Wallis univariate ANOVA (k samples) test was used for data comparison among multiple groups. *P* value was obtained from a bilateral test, ** *P* < 0.01, *** *P* < 0.001.

## Discussion

DN is a chief complication of diabetes and a leading cause of end-stage renal disease over the world [9]. Epidemiological data show that about 40% of diabetic patients will progress to DN, and podocyte injury is one of the main clinicopathological features [38]. TP is the major active component of Hook F, which has obvious immunosuppressive, anti-inflammatory, and podocyte-protective effects [9]. In this paper, we mainly elucidated that TP inhibited OS and inflammatory injury through the miR-155-5p/BDNF pathway, thus alleviating podocyte injury in DN.

The integral role of podocyte injury in DN has been reported [39]. TP can alleviate podocyte-associated glomerular diseases [40]. To explore the mechanism of TP on DN, we established the DN mouse models through HFD feeding and injection of STZ and then treated DN mice with TP for 12 weeks. After TP treatment, the fasting glucose and 24 h UMA of mice were decreased, the morphological changes of mouse kidney tissues and pathological changes of podocytes were improved, and Nephrin expression was increased. Consistently, TP can reduce proteinuria and podocyte injury in DN model animals [8,9], downregulated the genes essential for podocyte structure and function, and attenuated proteinuria and podocyte death [41,42]. Taken together, TP can improve DN and reduce podocyte damage in mice. In addition, we established a model of podocyte injury induced by HG *in vitro*, followed by TP treatment. DN is closely related to OS and inflammatory factor imbalance [1,2]. We determined the ROS levels, OS-related oxidase levels such as MDA, SOD, and GSH, and inflammation-related cytokines IL-1β, IL-6, TNF-α, and IL-4 in mouse podocytes and discovered that the OS levels and inflammation were up-regulated in HG mice but down-regulated after TP intervention. Moreover, TP had better improvement effects on the OS and inflammation of MPC5 cells better than Irbesartan. Previous research has elucidated the property of TP in repressing OS and inflammation [36,37]. Altogether, TP can inhibit OS injury and inflammatory injury of mouse podocytes induced by HG.

miRNAs are gradually becoming the important medium in the pharmacological activity of TP [43]. The overexpression of miR-155-5p in serum or plasma of DN patients is predicted to be a potential diagnostic marker for DN [14,15]. We detected the level of miR-155-5p in kidney tissues of mice and HG-induced MPC5 cells and found that miR-155-5p was overexpressed, while TP could inhibit its expression. Existing evidence reported that TP treatment can reduce the miR-155-5p expression in microglia [44]. TGF-β1-induced podocyte injury is closely related to an elevated miR-155 level and stimulated inflammatory responses [41,42]. These reports strongly support our conclusion that TP could inhibit miR-155-5p.

To identify the effect of miR-155-5p on podocyte injury, we overexpressed miR-155-5p in MPC5 cells treated with HG and TP and examined the OS and inflammation-related factors in MPC5 cells. Interestingly, overexpression of miR-155-5p reversed the protective effect of TP on injured mouse podocytes. Previous studies have elucidated that overexpression of miR-155 could promote the production of inflammatory molecules in podocytes, thereby aggravating podocyte injury [45,46]. Overexpression of miR-155-5p can reverse the protective effect of lncRNA CTBP1-AS2 in HG-stimulated human glomerular mesangial cells [47]. In short, TP alleviated OS and inflammatory damage in HG-induced MPC5 cells by inhibiting miR-155-5p.

BDNF is vital in the repair of podocyte injury in DN and the regulation of cellular OS and inflammation [19,22]. First, we confirmed the targeting relationship between miR-155-5p and BDNF through dual-luciferase experiments. Besides, we found that BDNF was down-regulated in DN mice and HG-induced MPC5 cells, but its expression was up-regulated after treatment with TP, and downregulated again after overexpression of miR-155-5p. It has been documented that miR-365 regulates STZ-induced DN fibrosis by regulating the BDNF-TRKB axis in renal function [20]. In conclusion, miR-155-5p targeted BDNF. To further explore the role of BDNF in mouse podocytes, we co-transfected miR-155-5p mimics and BDNF overexpressed plasmids into MPC5 cells treated with HG and TP. Expectedly, overexpression of BDNF alleviated OS and inflammatory injury and partially restored the miR-155-5p overexpression-inhibited protective effect of TP. There is evidence to suggest that BDNF participates in the regulation of inflammatory factors in HK-2 cells [20]. BDNF repairs podocyte injury by increasing actin polymerization and alleviating proteinuria and glomerular lesions [48]. As a whole, TP up-regulated BDNF by inhibiting miR-155-5p, thus inhibiting OS and inflammatory damage and alleviating podocyte injury induced by HG in mice.

In conclusion, TP reduced OS and inflammatory damage in DN mice based on the miR-155-5P/BDNF axis. This study provides a new insight for TP intervention in the treatment of DN and podocyte injury. However, limited by research conditions, there is a lack of clinical studies on the regulatory role of miR-155-5p in DN. Meanwhile, due to time constraints, we are not able to supplement the positive control group of treatment drugs in animal experiments. In future studies, positive controls of therapeutic drugs in animal experiments will be studied. Moreover, we will study the regulation of multiple miRNAs, target genes, and pathways in DN based on cell studies, which is of great significance for the pathogenesis of DN and gene-targeted therapy.

## Supplementary Material

Supplemental Material

## Data Availability

The data that support the findings of this study are available from the corresponding author upon reasonable request.
